This article has been retracted.

# Corydalis decumbens Can Exert Analgesic Effects in a Mouse Neuropathic Pain Model by Modulating MAPK Signaling

**DOI:** 10.1155/2022/7722951

**Published:** 2022-05-27

**Authors:** Yunting Chen, Zongbin Jiang, Aimin Zhang, Ruilin He, Zenghua Zhou, Shengrong Xu

**Affiliations:** ^1^Department of Pain Management, The Affiliated Hospital of Guizhou Medical University, Guiyang, 550004 Guizhou, China; ^2^Department of Pain Management, The Second Affiliated Hospital of Guangxi Medical University, 166 DaXue East Road, Nanning, 530007 Guangxi, China

## Abstract

**Objectives:**

This study is aimed at investigating the analgesic effect of the administration of Corydalis decumbens (CD) in a mouse model of postherpetic neuralgia (PHN) and at elucidating its mechanism of analgesic action.

**Methods:**

Adult Kunming (KM) mice were randomly divided into control, CD, and vehicle-treated groups. Neuropathic pain was induced with a single intraperitoneal injection of resiniferatoxin (RTX). Thermal hyperalgesia was assessed with a hot/cold plate test, and mechanical allodynia was evaluated using von Frey filaments. The activation states of astrocytes, microglia, and the mitogen-activated protein kinase (MAPK) pathway in the spinal cord were determined by immunofluorescence staining and Western blot analysis of Iba-1, GFAP, phospho-p38, and phospho-Jun N-terminal kinase (JNK).

**Results:**

RTX diminished thermal sensitivity and gradually increased sensitivity to tactile stimulation. The expression of Iba-1, GFAP, phospho-p38 MAPK, and phospho-JNK was upregulated in the RTX-induced postherpetic neuralgia mouse model. Systemic treatment with CD significantly ameliorated thermal sensitivity and mechanical hyperalgesia and was accompanied by a reduction in the expression of Iba-1 and GFAP and reduced phosphorylation of p38 and JNK.

**Conclusions:**

This study suggests that CD is effective at ameliorating mechanical hyperalgesia in PHN mice and that its mechanism of action may involve modulation of MAPK phosphorylation and glial cell activation. Thus, CD may be a promising alternative therapy for PHN.

## 1. Introduction

The rhizome of Corydalis decumbens Pers. (CD, named “Xiatianwu” in Chinese, family Papaveraceae) has been used as a Traditional Chinese Medicine (TCM) for the treatment of hemiplegia, hypertension, sciatica, and rheumatic arthritis, and it is officially listed in the Chinese Pharmacopoeia. Prior research has confirmed that alkaloids are the main active ingredients in CD, including protopine, tetrahydropalmatine, palmatine hydrochloride, and bicuculline [1]. Preinjection of protopine has been suggested to restrain the production of proinflammatory cytokines [2, 3] and also alleviate hydrogen peroxide-induced oxidative stress and apoptosis. Pretreatment with protopine can increase cell viability; improve the antioxidant activities of superoxide dismutase, catalase, and glutathione peroxidase; and reduce malondialdehyde levels in PC12 cells that have been injured with H_2_O_2_ [4]. Furthermore, tetrahydropalmatine possesses antihyperalgesic properties by reinforcing dopamine D1 receptor-mediated dopaminergic transmission [5], and the spatial learning and memory impairment that are induced by repeated administration of methamphetamine could be reversed by tetrahydropalmatine [6, 7]. Although the analgesic effect and anti-inflammatory bioactivity of many alkaloids derived from the rhizome of CD have been investigated, little research has been conducted to describe in detail the mechanism underlying the analgesic effect of CD injections to treat pain.

Postherpetic neuralgia (PHN) is a neuropathic pain syndrome resulting from a severe complication of herpes zoster infection [8]. Patients with PHN often exhibit profound mechanical allodynia and impairment of thermal sensitivity [9, 10]. While mechanical allodynia and hyperalgesia can be induced by an inoculation with varicella zoster virus or herpes simplex virus type 1 on the hind paw of rats or mice, the viral infection models are often incapable of inducing thermal impairment and have the shortcoming of developing tissue inflammation, skin lesions, and paralysis through spreading of the virus in the central nervous system [11–13]. Previous studies have demonstrated that systemic treatment with resiniferatoxin (RTX), an ultrapotent transient receptor potential vanilloid 1 (TRPV1) agonist, generates long-lasting paradoxical changes in thermal and mechanical sensitivities and can replicate the unique clinical symptoms of patients with PHN [14, 15]. Therefore, intraperitoneal injections of RTX have been used as a nonviral PHN model to explore new treatments that may effectively control this chronic pain condition [16, 17].

Activation of glial cells throughout the central nervous system, which comprise the spinal cord and cortex, and hyperactivation of proinflammatory mediators or neuropeptides are known to be critical in mediating neuropathic pain [18–21]. The mitogen-activated protein kinases (MAPK) are a family of serine/threonine protein kinases that consist of three primary members: extracellular signal-regulated kinase (ERK1/2), p38 mitogen-activated protein kinase (p38), and c-Jun N-terminal kinase (JNK). Many studies suggest that phosphorylation of p38, ERK, and JNK plays a significant role in neuropathic pain [22–25], and therefore, inhibition of the p38 MAPK pathway and/or activation of spinal microglia may be a potential therapeutic target for the treatment of cancer-induced bone pain [22]. Increased ERK, JNK, and p38 activation was demonstrated in a rat model of noncompressive lumbar disk herniation [26]. MAPK phosphorylation in the spinal cord regulates the intracellular responses that drive different downstream signaling events in neuropathic pain [27, 28]. The anti-inflammatory effect of protopine, an alkaloid derived from CD, can inhibit the phosphorylation of MAPK and the activation of NF-*κ*B [3].

This study investigated whether injections of CD could produce antinociceptive effects in a PHN mouse model that was induced by an intraperitoneal injection of RTX. The study further explored the mechanisms underlying CD-mediated antinociception and focused on the involvement of astrocytes and microglia and the activity of the p38 and JNK signaling pathways in the spinal cord. Our findings indicate that injections of CD can regulate the pain threshold by limiting the activation of microglia and astrocytes and by reducing the phosphorylation of JNK and p38 MAPK pathway components in the spinal cord.

## 2. Materials and Methods

### 2.1. Animals

Adult male Kunming (KM) mice (body weight, 18~22 g) were housed under a regular light-dark cycle in standard transparent plastic cages with *ad libitum* access to food and water. All handling procedures were approved and reviewed by the Guizhou Medical University (NO.1800959) and conducted in accordance with the guidelines of the International Association for the Study of Pain.

### 2.2. Experimental Design and PHN Model

Adult KM mice were randomly divided into three groups according to the random number table: control, CD, and vehicle-treated groups (20 per group). The PHN model was utilized in mice for the CD and vehicle-treated groups. Each mouse in the CD and vehicle-treated groups received a single intraperitoneal injection of RTX (50 *μ*g/kg, Sigma, St. Louis, MO), which was dissolved in a mixture of 10% Tween-80 and 10% ethanol in normal saline [29]. The control group received an equal volume of normal saline. According to the dose-to-dose relationship between humans and animals, the CD group was administered daily intraperitoneal injections of 120 *μ*g/kg of CD (Z36020694) in 2 mL of solution that contained protopine (0.4 mg/branch, JiangXi Herbi-sky Co., Ltd.) beginning 1 week after the RTX injection and lasting for 2 weeks. The vehicle-treated group received an equal volume of vehicle (normal saline containing 10% Tween-80 and 10% ethanol). The experimental design and process are shown in Figure 1(a).

### 2.3. Nociceptive Behavioral Tests

The behavior tests included mechanical (von Frey filament test) and thermal (hot-plate test) responses. Tests were assessed on the 1st day (T0) before RTX injection and the 1st (T1), 3rd (T2), 5th (T3), and 7th days (T4) after RTX administration and the 1st (T5), 3rd (T6), 5th (T7), 7th (T8), and 14th days (T9) after the initiation of CD injections. All tests were performed blinded to the groups and were conducted during the light phase. All mice were habituated to the testing environment for 30 min before assessment, during which time the exploratory and grooming activities were terminated.

#### 2.3.1. Hot-Plate Test

Thermal hyperalgesia was measured according to the methods described by Li et al. [30]. The hot-plate (IITC, USA) test was implemented at a constant temperature of 55 ± 0.5°C. The mice were enclosed in a plexiglass cage. The paw withdrawal thermal latency to thermal stimulation response (biting or licking hind paws or jumping) was recorded. Each test consisted of three independent trials separated by 30 min intervals. The mean latency for each mouse was calculated. A cutoff of 60 s was used to avoid potential tissue damage.

#### 2.3.2. Von Frey Filament Test

Mechanical allodynia was assessed using von Frey filaments (Stoelting, USA) by placing mice on an elevated wire mesh platform, and the paw withdrawal mechanical threshold (PWMT) was evaluated following application of von Frey filaments to the hind paw [27]. The test was initiated using a 1.0 g filament and ranged from 0.07 to 6 g, depending on the response (decreasing the strength after a positive response and increasing it after a negative response). The stimulation time was less than 5 s, with minimal intervals of 5 min. Biting, rapid pulling back, or shaking of the hind limb during or just after the stimulus was taken as a positive reaction.

### 2.4. Immunofluorescence

At two time points, one before the T4 CD injection and one after the last (T9), nociceptive behavioral responses were measured (T9). The mice were anesthetized with 2% sodium pentobarbital (20 mg/kg) and perfused transcardially with 50 mL of sterilized saline, followed by 100 mL of freshly prepared cold 4% paraformaldehyde in 0.1 M phosphate-buffered saline, (pH 7.4). The L4–L6 segments of the spinal cord were removed and postfixed in 4% paraformaldehyde, and the fixed samples were dehydrated, embedded in paraffin, and sectioned (3 *μ*m thickness, Leica, USA) [27, 31]. The slides were rehydrated, and antigen retrieval was performed prior to immunohistochemical staining. Slides were rinsed with PBS and incubated in a blocking buffer containing 0.3% Triton™ X-100 and 5% normal serum from the same species as the secondary antibody, in 0.1% PBS for 1 h at room temperature. Slides were then incubated with primary mouse anti-GFAP antibody (1 : 300, #3670, Cell Signaling Technology) and rabbit anti-Iba1 antibody (1 : 50, #019-19741, Wako Pure Chemical Industries, Osaka, Japan) for 24 h at 4°C. This incubation was followed by the addition of the corresponding secondary antibodies that were conjugated with Alexa Fluor®: 488-labeled goat anti-rabbit IgG (1 : 250) and 555-labeled Donkey anti-mouse IgG (1 : 250) in a dark chamber for 1 h. Finally, the sections were washed with PBS, a coverslip was applied, and stained sections were examined. Photographs were obtained under a fluorescent microscope (OLYMPUS, Japan), and both the intensities and areas of Iba1 and GFAP staining were measured using the ImageJ software (NIH, Bethesda, USA).

### 2.5. Western Blotting

Animals were decapitated under anesthesia with 2% sodium pentobarbital (20 mg/kg), and the L4-L6 spinal cord was quickly removed and homogenized in RIPA lysis buffer containing protease and phosphatase inhibitors. Total protein was extracted, and protein concentrations were quantified using a BCA Protein Assay Kit (70-PQ0012, MultiSciences Biotech Co., Ltd., China). A 20 *μ*g of total protein from each sample was loaded onto each lane, separated by 12% SDS-PAGE, and then transferred to a PVDF membrane in transfer buffer containing methanol. The membranes were blocked with 5% nonfat dry milk for 1 h, washed in Tris-buffered saline containing 0.1% Tween-20 (TBST), and then incubated with the following primary antibodies overnight at 4°C: rabbit anti-p38 MAPK antibody (1 : 1000, #8690T, Cell Signaling Technology), rabbit anti-phospho-p38 MAPK antibody (1 : 1000, #4511, Cell Signaling Technology), rabbit anti-SAPK/JNK antibody (1 : 1000, #9252T, Cell Signaling Technology), mouse anti-phospho-SAPK/JNK antibody (1 : 2000, #9255, Cell Signaling Technology), and anti-GAPDH antibody (1 : 20000, PTG). The membranes were washed with TBST and incubated with anti-rabbit or anti-mouse HRP-conjugated secondary antibodies for 1 h. Subsequently, the immunoreactive bands were detected using an ECL reagent (LK-P1421, MultiSciences Biotech Co., Ltd., China), and the intensities of the protein bands were measured by densitometry using the ImageJ software.

### 2.6. Statistical Analysis

Results are expressed as the mean ± SEM ($\bar{x}\pm s$). The behavioral data were analyzed by an ANOVA test followed by a Bonferroni test as a multiple comparison analysis. Alteration of the expression of the proteins detected was analyzed using a one-way ANOVA, followed by a Bonferroni test. Differences were considered to be statistically significant based on a criterion of *P* < 0.05.

## 3. Results

### 3.1. CD Administration Ameliorated RTX-Induced Neuropathy

PWMT and thermal latency were determined at T0-T9. Prior to RTX injections, there were no significant differences in both PWMT and thermal latency among the three groups at T0 (Figures 1(b) and 1(c), *P* > 0.05). From T1 to T4, RTX induced a significant decrease in PWMT and increase in thermal latency in the CD and vehicle-treated groups, compared with the control group (*P* < 0.05). From T6 to T9, intraperitoneal injections of 120 *μ*g/kg CD significantly ameliorated the mechanical hypersensitivity and decreased the withdrawal thermal latency compared with the vehicle group (*P* < 0.05).

### 3.2. CD Administration Significantly Reduced the Expression of GFAP and Iba1 in RTX-Induced PHN Mice

Immunofluorescence was utilized to identify changes in GFAP and Iba1 expression in the ipsilateral L4–L6 spinal cord. Previous research has shown that microglia and astrocytes are rapidly activated in the RTX-induced neuropathic pain models [9]. In this investigation, immunofluorescent images substantiated that these intraperitoneal injections of RTX significantly increased GFAP and Iba1 immunoreactivity in the spinal cord compared to the control group (*P* < 0.05). Compared to T4, protein levels of GFAP and Iba1 were significantly decreased in the CD treatment group at T9 (*P* < 0.05), but not in the vehicle group. These data suggest that RTX significantly stimulated microglia and astrocyte activation. Intraperitoneal administration of CD prominently inhibited RTX-induced astrocyte and microglia activation, as treatment with vehicle after RTX injection did not prevent activation (Figure 2).

### 3.3. Treatment with CD Effectively Attenuated p38 and JNK Phosphorylation in the Spinal Cord of RTX-Induced PHN Mice

Prior studies have confirmed that JNK and p38 MAPK activities promote the initiation and maintenance of neuropathic pain [23, 32]. These kinases are activated by phosphorylation. Western blotting was utilized to investigate if the administration of CD modulated the phosphorylation state of these two proteins. Western blotting demonstrated that RTX injections significantly increased the amount of phospho-JNK and phospho-p38 MAPK in L4-L6 spinal cord at T4 compared to the control group (Figure 3, *P* < 0.05). Following treatment with CD, the phosphorylation of p38 and JNK in the spinal cord was significantly reduced at T9 compared with T4. The expression levels of phospho-JNK and phospho-p38 were not changed in the vehicle group at T9 compared with T4. Therefore, these data suggest that intraperitoneal therapy with CD can attenuate RTX-induced phosphorylation of JNK and p38 MAPK (Figure 3).

## 4. Discussion

In this study, we investigated the mechanism of action of CD in a mouse model of postherpetic neuralgia and its potential use as a treatment for neuropathic pain. Behavioral testing indicated that CD administration improved thermal perception and alleviated mechanical allodynia in RTX-induced neuropathy. Furthermore, treatment with CD also suppressed the activation of microglia and astrocytes and significantly attenuated the expression of phospho-JNK and phospho-p38. Taken together, this study suggests that the analgesic effect of CD is in part due to the suppression of GFAP and Iba-1 expression, as well as downregulation of p38 and JNK phosphorylation in the spinal cord.

Neuropathic pain is a common form of chronic pain that is associated with peripheral and central nerve injury and is characterized by spontaneous pain, hyperalgesia, allodynia, and paresthesia [33]. PHN is a common category of neuropathic pain that can persist for months to years and negatively affects the quality of life and activities of daily life [34, 35]. Its clinical treatment is challenging due to the limited efficacy and severe side effects of conventional analgesics such as opioids, tricyclic antidepressants, anticonvulsants, and nonsteroidal anti-inflammatory drugs [35]. As a TCM, CD has anti-inflammatory and analgesic effects and is currently used in the treatment of rheumatoid arthritis [36, 37]. The alkaloids in CD, such as protopine and tetrahydropalmatine, can also attenuate hyperalgesia and suppress an inflammatory response [2, 38, 39]. Our current research evaluated the antinociceptive effects of CD in RTX-induced PHN mice.

In recent years, our understanding of PHN has centered on the action of neurotransmitters and ion channels. More recently, the critical importance of glial cells in the initiation and maintenance of neuropathic pain has become apparent [27, 40]. Activated spinal cord glia have been observed in neuropathic pain models, including in the presence of inflammation, nerve injury, and cancer [22, 41, 42]. There is evidence that astrocytes and microglia are activated in the etiopathogenesis of RTX-induced neuropathic pain. Treatment with the glial inhibitors minocycline and fluorocitrate attenuated nociceptive hyperalgesia and the expression of glial cell-related proteins [9]. In addition, in a bone cancer pain model, the natural polyphenol morin attenuated mechanical hyperalgesia and free movement pain by inhibiting the expression of GFAP in the spinal cord [43]. The elevated expression of Iba-1 and OX-42 in diabetic rats significantly declined with intrathecal injections of minocycline, with mechanical allodynia and thermal hyperalgesia also being attenuated [44]. The present investigation demonstrates that the systemic administration of CD could inhibit RTX-induced activation of microglia and astrocytes in the spinal cord and thus attenuate thermal hyperalgesia and mechanical allodynia in mice.

One possible intracellular mechanism that may be correlated with glial cell activation in neuropathic conditions is MAPK pathway activation. Previous studies have demonstrated that JNK phosphorylation in astrocytes and p38 phosphorylation in microglia may be involved in modulating pain conduction in neuropathic states [27]. In chronic constriction injury-induced neuropathic pain models, phosphorylated ERK1/2 and p38 MAPK are elevated [45], and phosphorylation of JNK signaling pathway components participated in pain signal transduction in astrocytes [46]. Furthermore, intraperitoneal injection of RTX leads to the upregulation of p38 MAPK, and treatment with fluorocitrate and minocycline can relieve nociceptive behaviors and reduce p38 expression [9]. Western blotting and immunofluorescence analysis in this study revealed that RTX enhanced the expression of phospho-p38 and phospho-JNK in the spinal cord. The administration of CD dramatically suppressed the expression of phospho-JNK and phopsho-p38.

This study utilized an RTX-induced neuropathic pain model to explore the antinociceptive effects of CD. The study evaluated pain behavior utilizing hot-plate and von Frey tests. The results revealed that significant analgesic effects began on the third day (T6) after treatment with CD. Suppression of glial cell activation and reduced phosphorylation of p38 MAPK and JNK may be strongly related to the potential clinical benefits of CD administration for reducing neuropathic pain.

## 5. Conclusion

In summary, this study has unveiled a novel direction for the potential treatment of postherpetic pain. The administration of CD significantly alleviated neuropathic pain, attenuated mechanical hypersensitivity, and improved the thermal sensitivity that was induced by RTX. This investigation suggests that the analgesic effect of CD may be associated with glial cells (astrocytes, microglia), p38 MAPK, and JNK. Therefore, CD is a promising candidate for use as a therapeutic analgesic agent.

## Figures and Tables

**Figure 1:** Administration of Corydalis decumbens reverses mechanical allodynia and thermal hyperalgesia. (a) Detailed timeline for the research program. Nociceptive behavioral tests were conducted on the 1st day before RTX injection and on the 1st, 3rd, 5th, and 7th days after RTX injection and on the 1st, 3rd, 5th, 7th, and 14th days after the administration of CD. The immunofluorescence and Western blot experiments were conducted before the CD injection treatment and after the last nociceptive behaviors were measured. (b, c) The administration of Corydalis decumbens attenuates mechanical allodynia and thermal hyperalgesia in a mouse model of neuropathic pain. ^∗^*P* < 0.05 compared to the control group; ^#^*P* < 0.05 compared with T4.

**Figure 2:** Corydalis decumbens decreases RTX-induced microglial and astrocyte activation in the spinal cord. Immunofluorescence results are expressed as fold changes relative to the control group at T4. (a) GFAP and (c) Iba1, representative photomicrographs of spinal cord sections in the control, vehicle, and CD groups. Image analysis data for GFAP (b) and Iba1 (d). Data are presented as the mean ± SD. ^∗^*P* < 0.05 compared with T0; ^#^*P* < 0.05 compared with T4.

**Figure 3:** Corydalis decumbens suppresses the phosphorylation of p38 and JNK in the spinal cord. Western blots are expressed as fold changes relative to the control group at T4. (a, c) Western blots indicate that the expression of p-p38/p38 relative to the control was increased in the vehicle and CD groups after injection of RTX at T4, which was significantly inhibited by Corydalis decumbens. (b, d) Western blots indicate that the expression relative to the control was increased in the vehicle and CD groups after injection of RTX. When treated with CD, the expression of p-JNK/JNK was decreased in the CD group. Data are presented as the mean ± SD. ^∗^*P* < 0.05 compared with T0; ^#^*P* < 0.05 compared with T4.

## Data Availability

The data used to support the findings of this study are available from the corresponding author upon request.

## References

[1] Shen Y., Han C., Jiang Y., Zhou X., Zhu Z., Lei X. (2011). Rapid quantification of four major bioactive alkaloids in *Corydalis decumbens* (Thunb.) Pers. by pressurised liquid extraction combined with liquid chromatography-triple quadrupole linear ion trap mass spectrometry. *Talanta*.

[2] Bae D. S., Kim Y. H., Pan C. H. (2012). Protopine reduces the inflammatory activity of lipopolysaccharide-stimulated murine macrophages. *BMB Reports*.

[3] Alam M. B., Ju M. K., Kwon Y. G., Lee S. H. (2019). Protopine attenuates inflammation stimulated by carrageenan and LPS via the MAPK/NF-*κ*B pathway. *Food and Chemical Toxicology*.

[4] Xiao X. H., Liu J., Hu J. (2008). Protective effects of protopine on hydrogen peroxide-induced oxidative injury of PC12 cells via Ca^2+^ antagonism and antioxidant mechanisms. *European Journal of Pharmacology*.

[5] Zhou H. H., Wu D. L., Gao L. Y., Fang Y., Ge W. H. (2016). L-Tetrahydropalmatine alleviates mechanical hyperalgesia in models of chronic inflammatory and neuropathic pain in mice. *Neuroreport*.

[6] Cao G. F., Zhang Y., Zhu L. (2018). The inhibitory effect of levo-tetrahydropalmatine on the methamphetamine- induced spatial memory impairment in mice. *Neuroscience Letters*.

[7] Chen Y. J., Liu Y. L., Zhong Q. (2012). Tetrahydropalmatine protects against methamphetamine-induced spatial learning and memory impairment in mice. *Neuroscience Bulletin*.

[8] Forbes H. J., Bhaskaran K., Thomas S. L. (2016). Quantification of risk factors for postherpetic neuralgia in herpes zoster patients: a cohort study. *Neurology*.

[9] Lei Y. S., Sun Y.ʼ., Lu C.ʼ., Ma Z., Gu X. (2016). Activated glia increased the level of proinflammatory cytokines in a resiniferatoxin-induced neuropathic pain rat model. *Regional Anesthesia and Pain Medicine*.

[10] Zou J., Dong X., Li Y. (2019). Deep sequencing identification of differentially expressed miRNAs in the spinal cord of resiniferatoxin-treated rats in response to electroacupuncture. *Neurotoxicity Research*.

[11] Kuraishi Y., Sasaki A. (2014). Animal models and pharmacology of herpetic and postherpetic pain. *Current Topics in Behavioral Neurosciences*.

[12] Dalziel R. G., Bingham S., Sutton D. (2004). Allodynia in rats infected with varicella zoster virus--a small animal model for post-herpetic neuralgia. *Brain Research Reviews*.

[13] Takasaki I., Andoh T., Shiraki K., Kuraishi Y. (2000). Allodynia and hyperalgesia induced by herpes simplex virus type-1 infection in mice. *Pain*.

[14] Yuan X. C., Wu C. H., Gao F. (2017). Activation and expression of *μ*-calpain in dorsal root contributes to RTX-induced mechanical allodynia. *Molecular Pain*.

[15] Pan H. L., Khan G. M., Alloway K. D., Chen S. R. (2003). Resiniferatoxin induces paradoxical changes in thermal and mechanical sensitivities in rats: mechanism of action. *Journal of Neuroscience*.

[16] Li H. P., Su W., Shu Y. (2019). Electroacupuncture decreases netrin-1-induced myelinated afferent fiber sprouting and neuropathic pain through mu-opioid receptors. *Journal of Pain Research*.

[17] Hong B. H., Sun J., Zheng H. (2018). Effect of tetrodotoxin pellets in a rat model of postherpetic neuralgia. *Marine Drugs*.

[18] Ali U., Apryani E., Wu H. Y., Mao X. F., Liu H., Wang Y. X. (2020). Low frequency electroacupuncture alleviates neuropathic pain by activation of spinal microglial IL-10/*β*-endorphin pathway. *Biomedicine & Pharmacotherapy*.

[19] Yang H., Wu L., Deng H. (2020). Anti-inflammatory protein TSG-6 secreted by bone marrow mesenchymal stem cells attenuates neuropathic pain by inhibiting the TLR2/MyD88/NF-*κ*B signaling pathway in spinal microglia. *Journal of Neuroinflammation*.

[20] Yin Y., Park H., Lee S. Y. (2019). Analgesic effect of toll-like receptor 4 antagonistic peptide 2 on mechanical allodynia induced with spinal nerve ligation in rats. *Experimental Neurobiology*.

[21] Yang F., Luo W. J., Sun W. (2017). SDF1-CXCR4 signaling maintains central post-stroke pain through mediation of glial-neuronal interactions. *Frontiers in Molecular Neuroscience*.

[22] Liu M. J., Yao M., Wang H. (2017). P2Y_12_ receptor-mediated activation of spinal microglia and p38MAPK pathway contribute to cancer-induced bone pain. *Journal of Pain Research*.

[23] Qu Y. J., Jia L., Zhang X., Wei H., Yue S. W. (2016). MAPK pathways are involved in neuropathic pain in rats with chronic compression of the dorsal root ganglion. *Evidence-based Complementary and Alternative Medicine*.

[24] Zhou J., Lin W., Chen H., Fan Y., Yang C. (2016). TRESK contributes to pain threshold changes by mediating apoptosis via MAPK pathway in the spinal cord. *Neuroscience*.

[25] Guo C. H., Bai L., Wu H. H. (2016). The analgesic effect of rolipram is associated with the inhibition of the activation of the spinal astrocytic JNK/CCL2 pathway in bone cancer pain. *International Journal of Molecular Medicine*.

[26] Miao G. S., Liu Z. H., Wei S. X., Luo J. G., Fu Z. J., Sun T. (2015). Lipoxin A_4_ attenuates radicular pain possibly by inhibiting spinal ERK, JNK and NF-*κ*B/p65 and cytokine signals, but not p38, in a rat model of non-compressive lumbar disc herniation. *Neuroscience*.

[27] Zhang F. F., Morioka N., Abe H. (2016). Stimulation of spinal dorsal horn *β*2-adrenergic receptor ameliorates neuropathic mechanical hypersensitivity through a reduction of phosphorylation of microglial p38 MAP kinase and astrocytic c-jun N-terminal kinase. *Neurochemistry International*.

[28] Sanna M. D., Ghelardini C., Galeotti N. (2016). Blockade of the spinal BDNF-activated JNK pathway prevents the development of antiretroviral-induced neuropathic pain. *Neuropharmacology*.

[29] Hsieh Y. L., Chiang H., Lue J. H., Hsieh S. T. (2012). P2X3-mediated peripheral sensitization of neuropathic pain in resiniferatoxin- induced neuropathy. *Experimental Neurology*.

[30] Li J. C., Shen X. F., Meng X. L., Zhang Y., Lai X. R. (2011). Analgesic effect and mechanism of the three TCM-herbal drug-combination Tou Feng Yu pill on treatment of migraine. *Phytomedicine*.

[31] Segat G. C., Manjavachi M. N., Matias D. O. (2017). Antiallodynic effect of *β*-caryophyllene on paclitaxel-induced peripheral neuropathy in mice. *Neuropharmacology*.

[32] Chen Y., Li G. W., Huang L. Y. M. (2015). p38 MAPK mediates glial P2X7R-neuronal P2Y1R inhibitory control of P2X3R expression in dorsal root ganglion neurons. *Molecular Pain*.

[33] Costigan M., Scholz J., Woolf C. J. (2009). Neuropathic pain: a maladaptive response of the nervous system to damage. *Annual Review of Neuroscience*.

[34] Friesen K. J., Chateau D., Falk J., Alessi-Severini S., Bugden S. (2017). Cost of shingles: population based burden of disease analysis of herpes zoster and postherpetic neuralgia. *BMC Infectious Diseases*.

[35] Mallick-Searle T., Snodgrass B., Brant J. M. (2016). Postherpetic neuralgia: epidemiology, pathophysiology, and pain management pharmacology. *Journal of Multidisciplinary Healthcare*.

[36] Wang Q., Li Z., Yang Z. (2016). New alkaloids with anti-inflammatory activities from *Corydalis decumbens*. *Phytochemistry Letters*.

[37] Yu S. Y., Yu Z. A. (2013). Clinical observation of compound xiatianwu tablets in treatment of 120 cases with active rheumatoid arthritis. *Zhongguo Zhong Yao Za Zhi*.

[38] Guo Z. G., Man Y., Wang X. (2015). Levo-tetrahydropalmatine attenuates oxaliplatin-induced mechanical hyperalgesia in mice. *Scientific Reports*.

[39] Zhang M. Y., Liu Y. P., Zhang L. Y. (2015). Levo-tetrahydropalmatine attenuates bone cancer pain by inhibiting microglial cells activation. *Mediators of Inflammation*.

[40] Watkins L. R., Maier S. F. (2003). Glia: a novel drug discovery target for clinical pain. *Nature Reviews Drug Discovery*.

[41] Doyen P. J., Vergouts M., Pochet A. (2017). Inflammation-associated regulation of RGS in astrocytes and putative implication in neuropathic pain. *Journal of Neuroinflammation*.

[42] Lim H., Lee H., Noh K., Lee S. J. (2017). IKK/NF-*κ*B-dependent satellite glia activation induces spinal cord microglia activation and neuropathic pain after nerve injury. *Pain*.

[43] Jiang W., Wang Y., Sun W., Zhang M. (2017). Morin suppresses astrocyte activation and regulates cytokine release in bone cancer pain rat models. *Phytotherapy Research*.

[44] Sun J. S., Yang Y. J., Zhang Y. Z., Huang W., Li Z. S., Zhang Y. (2015). Minocycline attenuates pain by inhibiting spinal microglia activation in diabetic rats. *Molecular Medicine Reports*.

[45] Piotrowska A., Kwiatkowski K., Rojewska E., Makuch W., Mika J. (2016). Maraviroc reduces neuropathic pain through polarization of microglia and astroglia - evidence from *in vivo* and *in vitro* studies. *Neuropharmacology*.

[46] Cao J., Wang J. S., Ren X. H., Zang W. D. (2015). Spinal sample showing p-JNK and P38 associated with the pain signaling transduction of glial cell in neuropathic pain. *Spinal Cord*.

